RETRACTED

# MicroRNA-143 Targets Syndecan-1 to Repress Cell Growth in Melanoma

**DOI:** 10.1371/journal.pone.0094855

**Published:** 2014-04-10

**Authors:** Ruiya Li, Lingli Zhang, Lizhou Jia, Yan Duan, Yan Li, Jie Wang, Lidao Bao, Na Sha

**Affiliations:** 1 Department of Dermatology, Inner Mongolia People's Hospital, Hohhot, Inner Mongolia Autonomous Region, China; 2 Department of Pathology, Inner Mongolia People's Hospital, Hohhot, Inner Mongolia Autonomous Region, China; 3 Department of Pathology, The Affiliated People's Hospital of Inner Mongolia Medical University, Hohhot, Inner Mongolia Autonomous Region, China; 4 Department of Dermatology, The Affiliated Hospital of Inner Mongolia Medical University, Hohhot, Inner Mongolia Autonomous Region, China; 5 Department of Pharmacy, The Affiliated Hospital of Inner Mongolia Medical University, Hohhot, Inner Mongolia Autonomous Region, China; University of Connecticut Health Center, United States of America

## Abstract

Melanoma is the most aggressive type of skin cancer with a rapid progression and a limited efficiency of therapeutics. Recently, studies have identified some microRNAs playing important roles in the development of melanoma. Syndecan-1 (Syn-1), dysregulated in many cancers, plays important roles in tumor progression by controlling cell proliferation. In this study, we investigated whether microRNA-143 (miR-143) is involved in the regulation of Syn-1 and thus plays a functional role in melanoma. We found that miR-143 expression was significantly lower in melanoma tissues than in normal tissues and its low expression was closely related to clinical stages of melanoma. Further experiments showed that consistent with the inhibitory effects induced by knockdown of Syn-1, overexpression of miR-143 suppressed cell proliferation, promoted G1 phase arrest and induced apoptosis in melanoma. Downregulation of miR-143 apparently produced opposite effects. Combined treatment of miR-143 overexpression and Syn-1 knockdown induced remarkable synergistic effects, while reconstitution of miR-143-resistant Syn-1 reversed the inhibitory activity of miR-143. Moreover, miR-143 level was inversely correlated with Syn-1 expression in melanoma cells. miR-143 directly targeted the 3′-untranslated regions of Syn-1 mRNA and they were in the same Argonaute2 complex. Taken together, this study revealed a link between miRNA-143 and Syn-1 in the pathogenesis of melanoma. MiR-143 plays an important role in the regulation of cell growth in melanoma. Restoration of miR-143 expression may represent a promising and efficient therapeutic approach for targeting malignant melanoma.

## Introduction

Melanoma is one of the most frequently diagnosed tumors in western countries, with increasing incidence rate, high probability of developing invasive cancers and mortality [1]. For many years, although much progress has been made in understanding the initiation and progress of melanoma, it is still assumed to be refractory to the current therapeutic interventions and little improvement on the survival rate has been made [2], [3].

RETRACTED

Recent studies have reported that microRNAs (miRNAs), a class of small non-coding RNAs 21–25 nucleotides in length, are important in tumorigenesis [4], [5]. miRNAs are initially linked to tumorigenesis due to their dysregulated levels [6] and mature miRNAs exert effects by post-transcriptionally regulating target genes through the 3′-untranslated region (UTR) to induce mRNA degradation and inhibit mRNA translation [7]. Depending on their cellular contexts and target genes, miRNAs may function as tumor suppressors or oncogenes [8]. Among these miRNAs, miR-143 has been demonstrated to significantly decrease in multiple cancer types and play a role of tumor suppressor. For instance, loss of miR-143 was observed in bladder cancer, whereas enhanced expression of miR-143 induced growth suppression in bladder cancer cells through downregulation of ERK5 and Akt expression at translational level [9]. miR-143 was also downregulated in colorectal cancer and non-small-cell lung **cancer,** and inhibited cell invasion and migration by repressing MACC1 or CD44v3 expressions respectively [10], [11]. However, the role of miR-143 in the regulation of key genes and signaling pathways associated with melanoma remains largely unknown.

In this study, we aimed to investigate the expression of miR-143 in melanoma tissues and explore its effect on growth of melanoma cells and its downstream target. We confirmed the regulatory relationship between miR-143 and its new target gene, Syndecan-1 (Syn-1). We provided evidences that miR-143 could impede melanoma cell growth, at least partly by targeting Syn-1. Our findings provide further evidence for the implication of dysregulated miRNAs in melanoma, and miR-143 may serve as a molecular target for melanoma, which to date has a dismal outcome with limited therapeutic options.

## Materials and Methods

### Tissue samples

For the use of clinical materials for research purposes, prior approval was obtained from the Medical Ethics Committee of Inner Mongolia People's Hospital (IMP study ID H05-561025). The study was conducted according to the principles expressed in the Declaration of Helsinki. All samples were collected and analyzed with prior written, informed consent of the patients. Skin tissues were obtained from patients (40 male and 32 female) who underwent surgery at Department of Dermatology, Inner Mongolia People's Hospital from 2005 to 2010. The study was carried out in accordance with the institutional ethical guidelines and the use of human skin tissues was approved by the Medical Ethics Committee of Inner Mongolia People's Hospital (IMP study ID H05-561025). Skin tissues from 10 healthy volunteers (matched by gender and age) were collected as normal controls. All samples were freshly frozen in liquid nitrogen, and then stored at −80°C for further use.

RETRACTED

### Cell culture and transfection

Human melanoma cells lines, including A-375, 1205Lu, UACC903, CHL-1 and sk-mel-5, were purchased from American Type Culture Collection. Cells were maintained in RPMI-1640 medium (A-375, 1205Lu) or DMEM medium (UACC903, CHL-1 and sk-mel-5) respectively supplemented with 10% fetal bovine serum in a 37°C humidified atmosphere of 5% CO_2_.

Ectopic expression of miR-143 in cells was obtained by transfection with miR-143 mimics or inhibitors (50 nM) using Lipofectamine2000. Knockdown of Syn-1 was performed using Syn-1 siRNA (100 nM). Human cDNA encoding Syn-1 was constructed using pcDNA 3.0 vector and transfected into cells to induce Syn-1's reconstitution. Cells were plated in 6-well or 96-well plates and transfected for 24 h or 48 h. Transfected cells were used in further assays or RNA/protein extraction.

### RNA extraction and quantitative real-time PCR analysis

Total RNA was extracted from tissues or cells using Trizol reagent. For miR-143 expression, total RNA was reverse-transcribed using the Taqman miRNA reverse transcription kit and real-time PCR was performed using TaqMan Universal Master Mix II. For Syn-1 mRNA expression, total RNA was reverse-transcribed using PrimeScript RT reagent Kit and real-time PCR was carried out using SYBR green PCR master mix. U6 snRNA or GAPDH expression was used as an endogenous control respectively. Gene expression was measured in triplicate and data were processed using 2^−ΔΔ^CT method and normalized to control.

### Protein extraction and western blot analysis

Cells were lysed in RIPA buffer with protease inhibitors. Protein was subjected to a SDS-PAGE minigel, transferred onto PVDF membrane and blotted using anti-Syn-1 antibody followed by the HRP-conjugated secondary antibody. Signals were visualized using ECL Substrates. GAPDH served as the loading control.

### CCK-8 cell proliferation assay

Cell proliferation rates were measured using Cell Counting Kit-8. Briefly, 0.5×10^4^ cells/well were seeded in a 96-well plate for 24 h, transfected with the indicated miRNA or siRNA, and further incubated for 24 h, 48 h and 72 h respectively. CCK-8 reagent (10 μl) was added to each well at 1 h before the endpoint of incubation. OD450 nm value in each well was determined by a microplate reader.

RETRACTED

### Apoptosis assays

Apoptosis assays were performed using Annexin V apoptosis detection kit. Briefly, transfected cells were collected, washed with PBS and resuspended in binding buffer containing Annexin V-FITC and propidium iodide (PI). After 15 min of incubation at room temperature, samples were analyzed on a FACSalibur flow cytometer to determine rate of apoptosis. Experiments were performed in triplicates and at least three times independently.

### Cell cycle assay

PI staining was performed to analyze cell cycle distribution. Briefly, 1×10^6^ cells were fixed in 70% ethanol and resuspended in 1 ml of RPMI media containing 50 μg/ml PI and 0.5 μg of RNase A at 37°C for 30 min. Samples were analyzed on a FACSalibur flow cytometer and the data were evaluated using the ModFit software program.

### Luciferase reporter assays

The 3′-UTRs of Syn-1 were amplified by PCR using the following primers: 5′-GTACCGGAGAAAGTGCGCTGCGCCA-3′ and 5′-AGCTTGRGGAAGGCTCT GCACCCGC-3′. The PCR products were then inserted into pGL3-basic vector. Target site mutations were generated using the PCR products with the appropriate primers containing point substitutions. The sequences were verified by DNA sequencing. HEK293T cells were co-transfected with 0.1 μg reporter plasmid with 0.65 pmol miRNA mimics or control miRNA in 96-well plates. Luciferase activity was detected 48 h later using a dual-luciferase reporter assay system and normalized to Renilla activity.

### RNA immunoprecipitation

Cell lysates were prepared from transfected cells using lysis buffer containing protease inhibitors and Rnase inhibitors. Protein A+G sepharose was successively incubated with normal rabbit IgG for 2 h, Argonaute 2 antibodie (Ago2, 1∶200) or isotope control for 2 h, and then protein lysates overnight. RNA was exacted using Trizol reagent after stringent washing followed by detection of miR-143 and Syn-1 expression by real-time PCR assay.

### Statistical analysis

All values were expressed as mean ± SD and processed using the SPSS 13.0 software. Statistical significance was noted at P<0.05. Three independent experiments were performed. The differences among the groups were estimated by Student's t-test or one-way ANOVA. The Mann-Whitney U test and Spearman's correlation analyses were used to analyze the relationship between miR-143 expression and the clinical features of melanoma or Syn-1 expression.

## Results

### miR-143 is downregulated in melanoma tissues and associated with clinical stages

We first tested the expression of miR-143 by real-time PCR in 30 patients with melanoma of various tumor stages compared with their age/gender-matched normal controls. The result revealed that miR-143 was downregulated in 86.67% (26/30) of the melanoma tissue samples compared to their matched normal control tissues (Figure 1A, P<0.01). Then the expression of miR-143 was quantified in 10 normal skin tissues and 72 cases of melanoma samples. As shown in Figure 1, relative miR-143 expression decreased along with the clinical stages (Figure 1B), progression of T classifications (Figure 1C), N classifications (Figure 1D) and distant metastasis (Figure 1E).

RETRACTED

**Figure 1:** Decreased expression of miR-143 in both melanoma tissues and cell lines. (A) Mean expression of miR-143 in the human melanoma tissues and normal skin tissues. Correlation between miR-143 expression and clinical stages (B), T classification (C), N classification (D) and distant metastasis (E) in melanoma tissues and normal skin tissues. The bounds of boxes represent the lower and upper quartiles; lines within boxes and whiskers denote median and extremum respectively. (F) Mean expression of miR-143 in five melanoma cell lines and skin tissues pooled from 3 healthy individuals. (G) Expression of miR-143 was significantly enhanced by transfecting miR-143 mimics into sk-mel-5 cells. (H) Expression of miR-143 was significantly reduced by transfecting miR-143 inhibitor into A-375 cells. (**P<0.01)

### Effects of miR-143 on melanoma cell proliferation, cell cycle and apoptosis

miR-143 expression was measured in five melanoma cell lines first. The total five cell lines showed a significant lower level of miR-143 compared to the normal control skin tissue pooled from 3 healthy individuals (Figure 1F, P<0.01). Moreover, miR-143 expression was relatively higher in A-375 and lower in sk-mel-5, thus we chose to overexpress miR-143 in sk-mel-5 cells by transfecting hsa-miR-143 mimics (Figure 1G) and silence miR-143 in A-375 cells by transfecting hsa-miR-143 inhibitor (Figure 1H) respectively to evaluate the possible role of miR-143 in melanoma pathogenesis.

CCK-8 assay revealed that the increased expression of miR-143 induced significant inhibition on sk-mel-5 cell proliferation compared to scramble control (Figure 2A). Correspondingly, decreased expression of miR-143 significantly stimulated A-375 cell proliferation (Figure 2B). Distributions of cells within the stages of cell cycle were determined by flow cytometry. After treated with miR-143 mimics, sk-mel-5 cells showed a significant increased percentage of cells in the G1 peak and a decreased percentage of cells in the S and G2 peak (Figure 2C, P<0.01). However, A-375 cells treated with miR-143 inhibitor showed a dramatic decrease in the percentage of cells in the G1 peak and an increase in the percentage of cells in the S and G2 peak (Figure 2D, P<0.01). Moreover, the rate of apoptosis was significantly higher in sk-mel-5 cells with higher expression of miR-143 (Figure 2E, P<0.01) but was remarkably decreased when miR-143 was inhibited in A-375 cells (Figure 2F, P<0.01). Taken together, these results suggested that miR-143 could inhibit cell proliferation, repress cell cycle progression and promote apoptosis in melanoma cells.

RETRACTED

**Figure 2:** Effects of miR-143 on proliferation, cell cycle and apoptosis of sk-mel-5 and A-375 cells. (A, B) Cell proliferation analyzed by CCK-8 assays. (C, D) Flow cytometry analyses of cell cycle. (E, F) Flow cytometry analyses of cell apoptosis. Left panel and middle panel, flow cytometry analyses of various cells. Right panel, quantification of cell cycle population or apoptotic rate. Annexin-FITC positive cells were analyzed for apoptotic rate (Right low quadrant: early apoptotic rate, right high quadrant: late apoptotic rate). (**P<0.01, *P<0.05, Figure is representative of 3 experiments with similar results.)

### Correlation of expression between miR-143 and Syn-1

Using online miRNA target prediction databases (miRNA.org, Pictar and Targetscan), we hypothesized that Syn-1 was a target of miR-143 (Figure 3A). To confirm the relevance, we then investigated the expressions of Syn-1 in melanoma cells with altered expression of miR-143. Quantitative PCR showed that the mRNA levels of Syn-1 were dramatically downregulated in miR-143-overexpressing cells, whereas it was upregulated after inhibition of miR-143 (Figure 3B). Apparent alterations of Syn-1 protein expression were also observed by western blot analysis (Figure 3D). Then we examined the Syn-1 expression profile in melanoma cells. Both PCR and western blot analysis showed that all the five cells showed a notable high level of Syn-1 compared to the skin tissue pooled from 3 healthy individuals (Figure 3D and E). Moreover, an inverse correlation of expression between miR-143 and Syn-1 mRNA was observed (R = -0.8632, P<0.05, Figure 3F). These results suggested a potential regulation of Syn-1 by miR-143.

**Figure 3:** Negative correlation between miR-143 and Syn-1. (A) The predicted miR-143 binding site within Syn-1 3′UTR and its mutated version by site mutagenesis are as shown. (B, C) Upregulated expression of miR-143 inhibited Syn-1 expression at both mRNA and protein level, while reduction of miR-143 restored Syn-1 expression. (D, E) Variable Syn-1 expression in five melanoma cells and normal control skin tissues pooled from 3 healthy individuals. GAPDH was used as the loading control. (F) An inverse correlation was observed in five melanoma cells (Spearman's correlation, R = −0.8632). (**P<0.01, *P<0.05, Figure is representative of 3 experiments with similar results.)

RETRACTED

### Syn-1 is a direct target of miR-143

To experimentally identify regulation between miR-143 and Syn-1, we preformed RNA immunoprecipitation of Syn-1 from the Ago2 complex and Luciferase reporter assays. We first overexpressed miR-143 in sk-mel-5 cells and analyzed the mRNAs associated with Ago2 using co-immunoprecipitation based on the functional co-complex of Ago2 with miR-143 and its target mRNA. Quantitative PCR showed that after miR-143 was successfully enriched in cells overexpressing it (Figure 4A, B); Syn-1 mRNA binding to the co-complex was also significantly increased compared to the scramble control (Figure 4 C). To further investigate if the predicted binding site of miR-143 to 3′UTR of Syn-1 is responsible for the regulation, we subcloned the Syn-1 3′-UTR fragment containing one miR-143 binding site and the mutant fragment into the luciferase reporter vector. As shown in Figure 4D, the luciferase activity was significantly reduced in miR-143 transfected cells, but mutations in the tentative miR-143-binding region in Syn-1 3′-UTRs abrogated the miR-143-mediated repression of luciferase activity. These results demonstrated that miR-143 could directly target Syn-1.

**Figure 4:** miR-143 directly targets Syn-1. (A) Association of miR-143 and Syn-1 with Ago2. Cellular lysates from sk-mel-5 cells transfected with or without miR-143 mimics were used for RNA immunoprecipitation with Ago2 antibody. Detection of Syn-1 (B) and miR-143 (C) in the same RISC complex using real-time PCR. (D)The repression of luciferase activity by Syn-1 3′UTR was dependent on miR-143. Mutated Syn-1 3′UTR abrogated miR-143 mediated repression luciferase activity (**P<0.01, Figure is representative of 3 experiments with similar results.)

### Syn-1 plays a crucial role in miR-143-regulated cell proliferation, cell cycle arrest and apoptosis

To further confirm the functional relationship between miR-143 and its downstream gene Syn-1, we downregulated Syn-1 expression in miR-143-silencing A-375 cells by co-transfection of Syn-1 siRNA and miR-143 mimics, and tested their effects on cell proliferation, cell cycle and apoptosis. Once Syn-1 expression was effectively depressed by siRNA (Figure 5A), transfected A-375 cells exhibited decreased cell proliferation (Figure 5B), a modest cell cycle arrest (Figure 5C and E) and increased apoptosis rate (Figure 5D and F), which was consistent with the effects induced by upregulation of miR-143. When cells were treated with Syn-1 siRNA in combination with miR-143 mimics, synergistic effects on cell proliferation (Figure 5B), cell cycle (Figure 5C and E) and apoptotic rate (Figure 5D and F) were observed. Moreover, we reconstituted Syn-1 in pre-miR-143 transfected cells to explore whether Syn-1 could reverse the inhibitory activity of miR-143. The silenced expression of Syn-1 in A-375 cells induced by higher expression of miR-143 was significantly relieved app:addword:alleviateby Syn-1 transfection (Figure 5A). The subsequent changes of cell proliferation, cell cycle arrest and apoptosis were all rectified as well (Figure 5B-F). Taken together, these results directly indicated that miR-143 functions as a potent tumor suppressor through regulating Syn-1 expression.

RETRACTED

**Figure 5:** Functional effects of Syn-1 on sk-mel-5 cells with altered expression of miR-143. (A) Effectively suppression of Syn-1 protein expression by Syn-1 siRNA and miR-143 mimics respectively and combinedly. Suppression of Syn-1 significantly inhibited cell proliferation (B) and induced G1 phase arrest (C) and cell apoptosis (D). Note the synergistic inhibitory effect induced by combination of Syn-1 siRNA and miR-143 mimics, compared with either of them alone. Reconstitution of miR-143-resistant Syn-1 by Syn-1 plasmid reversed the above inhibitory activity of miR-143. (**P<0.01, *P<0.05, Figure is representative of 3 experiments with similar results.).

## Discussion

Recently, the crucial role for miRNAs in tumor development has been suggested by the identification of numerous miRNAs dysregulation, which can drive tumorigenesis as tumor suppressors or oncogenes in many types of tumors [12], [13]. There have been emerging researches suggesting that miRNAs play essential roles in the development and progression of melanoma [14]. For example, miR-26a directly targets Lin28B and Zcchc11 to inhibit tumorigenesis and strongly prevent spontaneous and distant melanoma metastasis [15]. Melanoma cell lines with ectopic miR-211 exhibit significant growth inhibition and reduced invasiveness, and the negative post transcriptional effects of miR-211 on KCNMA1 transcript is responsible for the tumor-suppressor activities of MITF and/or TRPM1 [16]. miR-203 had a pivotal anti-oncogenic role in melanoma through reducing melanosome transport and promoting melanogenesis by targeting kif5b and through negative regulation of the CREB1/MITF/Rab27a pathway [17]. However, as a known tumor suppressive miRNA, little expression or functional confirmation of miR-143 in melanoma was reported.

In the current study, we clearly showed that miR-143 was downregulated in melanoma tissues and correlated with clinical stages. We further confirmed miR-143 overexpression was able to inhibit growth in sk-mel-5 cells (predominantly low miR-143 expression), accompanied by an increase of cells arrested in the G1 phase and an induction of cell apoptosis. On the contrary, when miR-143 expression was silenced, A-375 cells (relatively high miR-143 expression) exhibited stimulated cell growth. These findings suggested that miR-143 was involved in the processes of development of melanoma.

RETRACTED

Syn-1, a member of type I transmembrane heparan sulfate proteoglycans expressed predominantly in epithelial cells, plays important roles in tumor progression, inflammation and wound healing by controlling cell proliferation, differentiation, adhesion and migration [18], [19]. Syn-1 expression is dysregulated in many cancers. High expression of Syn-1 can be found in bladder cancer, colorectal cancer and breast cancer and is associated with a worse prognosis [20], [21]. Syn-1 modulates a multitude of physiological processes relevant to tumor progression, such as cancer cell proliferation and apoptosis, angiogenesis and metastasis [22]. And Syn-1 is required for robust growth, vascularization, and metastasis of myeloma tumors [23]. So far, little is known about Syn-1 in melanoma, but it has been suggested that expression of Syn-1 on the melanoma cell surface and its degradation by heparanase are important determinants in the control of tumor cell invasion and metastasis [24]. Our results confirmed a vital molecular relationship between miR-143 and Syn-1. We showed that, at both mRNA and protein level, upregulation of miR-143 expression in sk-mel-5 cells effectively suppressed Syn-1 expression, while in A-375 cells, downregulation of miR-143 enhanced its expression. There was also an inverse correlation between them in melanoma cell lines. Furthermore, this potential relevance was verified by luciferase reporter study and RNA immunoprecipitation using antibody against Ago2, a key component of the RNA-induced silencing complex (RISC). miR-143 directly target Syn-1 through binding to specific complementary site within its 3′ untranslated region. By overexpressing miR-143, Ago2-bound Syn-1 mRNAs could be successfully co-immunoprecipitated, suggesting that both Syn-1 and miR-143 are likely in the same Ago2 complex. Loss-of-function study of Syn-1 by siRNA-mediated knockdown demonstrated suppressive effects on cell growth, which were also verified in study by enhanced miR-143 expression. Taken together, these findings sufficiently consolidated that miR-143 played a suppressive role in cell growth, at least, in part due to directly inhibiting Syn-1 expression.

The RAS/RAF/MAPK pathway is hyperactive in about 30% of human cancers and required in the regulation of cell proliferation, survival and differentiation. Aberrant regulation of MAPK cascades contribute to cancers including malignant melanoma and many other human diseases [25], [26]. Xu et al. [27] reported miR-143 played an important role in prostate cancer proliferation, migration and chemosensitivity by suppressing KRAS and subsequent inactivation of MAPK pathway. miR-143 is a critical regulator of cell cycle activity via transcriptional regulation of MAPK7 (ERK5) signaling [28] and MAPK1 (ERK2) could also be a direct target of miR-143 [29]. As to Syn-1, its overexpression had profound effects on genes including MAPK/ERK pathways, TGF-β, EGF and VEGF to regulate cell growth, cell cycle progression, adhesion and migration [30]. Syn-1 can also induce apoptosis in breast cancer through inhibition of MAPK/ERK/Bad signaling [31]. Consistent with the previous studies, our results revealed a synergistic inhibitory effect of upregulated miR-143 and downregulated Syn-1 on cell growth, and partly elucidated a potential molecular mechanism by which miR-143 participated in melanoma development.

RETRACTED

Recently, more and more diagnostic and prognostic algorithm is supported by molecular alterations at the miRNAs level. miRNAs represent potential biomarkers for cancer diagnosis, prognosis and therapy. Their application to body specimens from blood to tissues has been helpful for appreciating their use in the clinical context [32], [33]. Our results showed that miR-143 was commonly downregulated in melanoma patients, and this downregulation was associated with clinical characteristics of patients, suggesting miR-143 may be a new potential diagnostic factor and target of melanoma. Further investigation will be required to elucidate this question.

In conclusion, our findings suggest that miR-143 is downregulated in melanoma and affects cancer cell growth by targeting Syn-1. The miR-143/Syn-1 relationship provided a potential mechanism for Syn-1 dysregulation and melanoma cell growth. As a result, restoration of miR-143 expression could have an important implication for therapeutic approach for melanoma.
